The article "Auditory Event-Related Potentials Associated With Music Perception in Cochlear Implant Users" was published in 2018. Journal: Front Neurosci.

# Auditory Event-Related Potentials Associated With Music Perception in Cochlear Implant Users

**DOI:** 10.3389/fnins.2018.00538

**Published:** 2018-08-07

**Authors:** Andréanne Sharp, Audrey Delcenserie, François Champoux

**Affiliations:** ^1^École d'orthophonie et d'audiologie, Université de Montréal, Montreal, QC, Canada; ^2^Département de psychologie, Université de Montréal, Montreal, QC, Canada

**Keywords:** electrophysiology, cochlear implants, deafness/hearing loss, music perception, brain plasticity, cortical reorganization

## Abstract

A short review of the literature on auditory event-related potentials and mismatch negativities (MMN) in cochlear implant users engaged in music-related auditory perception tasks is presented. Behavioral studies that have measured the fundamental aspects of music perception in CI users have found that they usually experience poor perception of melody, pitch, harmony as well as timbre (Limb and Roy, 2014). This is thought to occur not only because of the technological and acoustic limitations of the device, but also because of the biological alterations that usually accompany deafness. In order to improve music perception and appreciation in individuals with cochlear implants, it is essential to better understand how they perceive music. As suggested by recent studies, several different electrophysiological paradigms can be used to reliably and objectively measure normal-hearing individuals' perception of fundamental musical features. These techniques, when used with individuals with cochlear implants, might contribute to determine how their peripheral and central auditory systems analyze musical excerpts. The investigation of these cortical activations can moreover give important information on other aspects related to music appreciation, such as pleasantness and emotional perception. The studies reviewed suggest that cochlear implantation alters most fundamental musical features, including pitch, timbre, melody perception, complex rhythm, and duration (e.g., Koelsch et al., 2004b; Timm et al., 2012, 2014; Zhang et al., 2013a,b; Limb and Roy, 2014). A better understanding of how individuals with cochlear implants perform on these tasks not only makes it possible to compare their performance to that of their normal-hearing peers, but can also lead to better clinical intervention and rehabilitation.

## Introduction

Listening to and playing music are pleasurable activities of everyday human life. However, in order to be able to enjoy music, a complex analysis of the musical excerpt has to be done by the peripheral and central auditory systems, which then elicits emotions and/or meaning.

In both normal-hearing and cochlear implant listeners, mismatch negativity (MMN) patterns in event-related neural electrical potentials can be used to assess basic auditory percpetual discriminations most critical for music perception (pitch, timbre, loudness as well as melodic, and rhythmic patterns). The MMN component is a deviant-minus-standard difference waveform that is computed by subtracting the averaged event-related potential waveofrm in response to a repeated “standard” stimulus from that produced by a different, rarely presented novel, “deviant” stimulus (oddball paradigm). In general, the MMN is a reliable neural marker for the perceptual contrast (discriminability) between the rare novel stimulus and the much more probable standard one (see Näätänen et al., 1978 for more details).

The article "Auditory Event-Related Potentials Associated With Music Perception in Cochlear Implant Users" was published in 2018. Journal: Front Neurosci.

More complex processes, such as pleasantness, emotions or meaning, usually associated with music, can be evaluated using electrophysiological measurements of cortical activations–including the N400 component or frontal alpha asymmetry correlates. The N400 component is an event-related potential associated with the meaning of a stimuli and, in the case of music, meaning corresponds to the ability to associate a concept with musical excerpts. One type of protocol used to elicit the N400 component is to compare a prime stimulus with a target stimulus. For example, a fast song that contains a lot of high frequencies is usually more closely associated with the concept of a mouse than that of an elephant. The closer the association between these two stimuli, the less negative the amplitude of the N400 will be. The other technique, namely, the frontal alpha asymmetry measurement, is a relatively recent technique that has been used to examine the perceived pleasantness of a stimulus. This protocol consists in placing electrodes on each side of the head over the frontal area in order to obtain an imbalance index (Maglione et al., 2015).

In contrast to their normal-hearing peers, deaf individuals need an auditory compensation device in order to access an auditory experience of music. The typical way to restore hearing is to insert electrodes in the cochlea to directly stimulate the auditory nerve. This process, called cochlear implantation, can convert a severe-to-profound sensorineural hearing loss into near-normal hearing. Although implants successfully provide access to speech perception, CI users usually complain about the fact that implantation impairs their perception of music—specifically in cases of acquired deafness (e.g., Limb and Roy, 2014). Behavioral studies have confirmed this by assessing basic aspects of music perception in CI users and showing that these listeners have very poor perception of pitch, melody, harmony, and timbre (Limb and Roy, 2014). However, their perception of rhythm is generally well preserved (e.g., McDermott, 2004; Looi et al., 2012).

The article "Auditory Event-Related Potentials Associated With Music Perception in Cochlear Implant Users" was published in 2018. Journal: Front Neurosci.

On the one hand, it is well known that the signals that individuals are able to perceive with implants are degraded—an important limitation that may contribute to music perception deficits mentioned above (for a review see Limb and Roy, 2014). The spectral resolution that can be conveyed through CIs is much reduced compared to spectral resolution in the normal hearing system. Also, the possible interaction between electrodes is a limiting factor, because it decreases the quantity of possible independent channels for conveying information. The characteristics of the implants are leading to a bad replication of place-coded information. Finally, another problem is that CIs are not replicating temporal firing patterns that are essential for the representation of musical pitch and spectral fine structure, resulting in a bad replication of temporally-coded information by CI users.

Furthermore, studies suggest that the prolonged period of auditory deprivation that deaf individual experience prior to implantation may lead to brain alterations. For example, research shows that deprivations experienced in a given sensory modality can lead to the reorganization of the sensory cortex associated with this modality, known as cross-modal plasticity (e.g., Bavelier and Neville, 2002; Good et al., 2014; Houde et al., 2016). Similarly, a recent neuroimaging study has found that, in deaf individuals, auditory regions are activated by vibrotactile stimuli (Schürmann et al., 2006). These studies indirectly suggest that the altered perception of music experienced by CI users is possibly due, in part at least, to this cross-modal plasticity.

To date, no review has looked specifically at the auditory event-related correlates associated with CI users' music perception. The main goal of the present short review was to examine these electrophysiological responses that can be really useful to better understand music perception in CI users. An emphasis will be put on studies that have examined perception of musical pitch, melody, harmony, timbre, rhythm, tempo, meter, duration, and intensity by using auditory event-related potentials.

Moreover, and as mentioned earlier, electrophysiological measurements, such as the N400, frontal asymmetry measurement, and the MMN, are useful to examine the complex processes associated with music perception in normal-hearing individuals. Similarly, using electrophysiological measurements in hearing-impaired individuals could be useful to investigate the causes of CI users' impaired music perception. Thus, a secondary goal of the present review was to investigate the electrophysiological markers that can be used to document CI users' impaired music perception. The present review will focus on two electrophysiological techniques that have been used to investigate music perception, that is, measurements of the pleasantness and of the meaning of music. Overall, the present review aims to help clinicians by allowing them to plan their interventions with CI users more effectively. Since music perception is often a priority of CI users, clinicians must be properly trained to offer them appropriate and efficient rehabilitation.

The article "Auditory Event-Related Potentials Associated With Music Perception in Cochlear Implant Users" was published in 2018. Journal: Front Neurosci.

### Perception of musical pitch, melody, and harmony

The present review will focus mainly on pitch perception and, to a smaller extent on melody. It is however important to highlight that it is pitch perception that makes it possible for people to have a good understanding of music harmony, thus explaining why so many studies have investigated this ability.

On the one hand, behavioral studies suggest that CI users' performance on tasks assessing pitch perception is generally poor because of factors related to the technological limitations of the implant, including the implant processor and the design of its electrode (see Limb and Roy, 2014 for a review).

A study by Zhang et al. (2013b) used electrophysiological measurements, specifically the MMN, in order to examine pitch perception patterns. They compared 10 CI users to 10 normal-hearing controls (NH) using four different oddball paradigms. The participants were either exposed to a sequence of five notes with a standard pitch contour pattern [4 conditions: pattern in which each note was separated by one semi-tone starting at 440 Hz (1) rising or (2) falling or by five semi-tone (3) rising or (4) falling] or to a deviant pitch contour pattern [4 conditions paired with the equivalent standard stimuli (rising-flat or falling-flat): the 3 first notes followed the pattern separated by one or five semi-tone, but the last two notes of the pattern were the same as the third]. The presence of an MMN in participants indicated that they were able to detect the change in pitch contour pattern. However, in the one semi-tone pitch contour paradigm, none of the CI users exhibited an MMN response. An MMN was found in 30% of the CI users and in 80% of the NH controls in the rising pitch condition, whereas, in the falling pitch condition, 60% of the CI users and 80% of the NH controls had an MMN. This suggests that individuals with CIs have more difficulty discriminating pitch contour patterns than their NH peers (see also Timm et al., 2014 for similar results).

The article "Auditory Event-Related Potentials Associated With Music Perception in Cochlear Implant Users" was published in 2018. Journal: Front Neurosci.

Studies have also investigated more complex musical features related to pitch perception, but these studies have used different electrophysiological paradigms. For example, Sandmann et al. (2009) examined pitch perception. To do so, they compared 12 CI users to 12 NH controls using an oddball design in two different conditions—a dyadic tonal interval condition and a passive listening condition. Dyadic tonal intervals consisted of two sinusoidal tones, sampled at 44.1 kHz and tuned to the equal-tempered chromatic scale in the range of A4 (440 Hz) and Eb6 (1,245 Hz). These simple tones were paired at pitch intervals of 1 (minor second) and 18 (minor duodecim) semitones, resulting in two different dyadic tonal intervals. During this task, they looked specifically at the elicitation of the N1 component. This component is usually elicited when an unpredictable stimulus is detected, suggesting that a change in the auditory stimulus has been perceived (in that case, a difference in pitch). The dyadic tonal intervals could be defined as a simple frequency relationship between two notes. Sequences of musical intervals are fundamental features that constitute melodies. The results showed that the CI users exhibited smaller N1 amplitudes over their fronto-central area as well as altered hemispheric asymmetries when required to process dyadic tones. Effectively, the results showed that CI users exhibit a contralateral dominance for right-ear stimulation, while NH individuals exhibit a contralateral dominance for left-ear stimulation.

Given that, as already mentioned, pitch perception makes it possible to understand music harmony, CI users' pitch perception difficulties reviewed in the electrophysiological and behavioral studies described above may explain why they have an impaired appreciation of music (see also Limb and Roy, 2014 for a review).

### Perception of timbre

An extensive number of behavioral studies show that CI users experience difficulties with timbre perception (for a review, see McDermott, 2004). Timbre is the set of auditory qualities that distinguishes two different instruments playing the same note (i.e., the same pitch). A task in which subjects have to identify musical instruments is thus a task that relies on timbre perception.

Electrophysiological studies, on the other hand, generally report that, in normal hearing individuals, music-syntactic irregularities elicit negative electric brain potentials (around 200 and 500 ms). These negative brain potentials include the early right anterior negativity (ERAN), the N5, the MMN, and the P3 components. In general, these components are elicited when an individual detects novel or deviant stimuli. For example, a study by Koelsch et al. (2004b) has used music-syntactic irregularities; a concept associated with pitch, and timbre deviation to compare CI users and NH individuals on EEG responses for different negative electric brain components—the ERAN, the N5, the MMN, and the P3 components. The participants included 12 CI users and 12 NH who were instructed to count the number of deviant instruments in a sample of 216 chord sequences that each consisted of five chords. Note that, here, a deviant instrument refers to an instrument that differs from the piano (in this experiment deviant instruments were: trumpet, organ and other instruments sample available). In each chord sequence, there was a 25% chance that the third chord was irregular (syntactic irregularities: expected elicitation of the ERAN and the N5), a 25% chance that the fifth chord was irregular (syntactic irregularities: expected elicitation of the ERAN and the N5), and a 15% chance that the chords two to five were played by another instrument (expected elicitation of the MMN and the P3). In terms of syntactic irregularities, there was a significant group difference was found for ERAN and N5 responses. For the CI group, the amplitude of both complexes was smaller, but only for the fifth chord irregularity. As well, no ERAN or N5 responses were found in the CI users when the third chord was irregular. However, the amplitude of CI users' response was significantly smaller, suggesting diminished neural responses to violations of harmonic expectancy. In CI users, the timbre deviation condition also elicited an MMN response that was smaller in amplitude than that of NH individuals (by a factor of three). The latter results are not only consistent with those reported in the previous section, namely that CI users experience altered pitch perception, but they also suggest that basic timbre perception is a weakness of CI users.

The article "Auditory Event-Related Potentials Associated With Music Perception in Cochlear Implant Users" was published in 2018. Journal: Front Neurosci.

More recently, Timm et al. (2012) focused on the perception of temporal features related to timbre. They used an oddball paradigm in which the length of the stimuli were either shortened, by cutting off the first 60 ms (referred to as shortened attack time), or prolonged (prolonged attack time) in comparison to a standard normal stimulus (a 360 Hz French horn sound). The authors also examined basic auditory features using evoked potentials, specifically N1 and P2 amplitudes as well as latencies. The N1-P2 complex is known to be associated with the encoding of the physical attributes of sound in normal hearing individuals, such as the detection of stimulus onset (Weise et al., 2012). They recruited 12 CI users and 12 NH controls. In both groups, some participants had some musical training while others did not. The groups were matched on age and gender. The results showed that, in the NH group, a significant MMN response was elicited when the stimulus was presented in the prolonged attack time, but no significant MMN response was measured for the shortened attack time. In contrast, no MMN response was elicited in the CI group—this for all conditions. An absence of MMN response suggests that individuals with CIs experience reduced timbre perception. In terms of the N1 response, two interesting findings were reported. First, it was found that the amplitude of the N1 response in the CI users was significantly smaller than that of the control. Second, the amplitude of N1 responses in the CI users with prior musical training was more similar to that of the normal-hearing controls (with and without musical training) than to that of the CI users without musical training. These results suggest that musical training has an important impact on hearing experience.

Similarly, Zhang et al. (2013a) used MMN responses to look at timbre discrimination in CI users and their NH peers. To do so, they used three different oddball paradigms in which CI users and NH controls heard a musical note played by three different pairs of musical instruments (i.e., saxophone/piano, cello/trombone, and flute/French horn). In this protocol, a sequence of repetitive standard stimuli (saxophone, cello or flute) was infrequently interrupted by a deviant stimulus (piano or trombone or French horn). An MMN response, evoked by the presentation of the deviant stimulus, was measured for each of the three different pairs of musical instruments. Interestingly, the CI users exhibited MMN peaks that were significantly smaller and shorter in terms of both amplitude and duration than those of the NH group. These results corroborate those of previous electrophysiological studies in showing that timbre discrimination is altered in CI's users (Koelsch et al., 2004b; Timm et al., 2012).

Although interesting, the studies described above have used a paradigm that is relatively simple in order to measure timbre perception, that is, the ability to discriminate between two musical instruments. Rahne et al. (2014) recently used a more complex paradigm to investigate timbre perception, namely, a multifaceted protocol. In contrast to the protocols described earlier, the multifaceted protocol is particularly innovative since it allows the investigation of both spectral and temporal aspects of timbre at the same time. This more complex protocol was created to show that MMN responses could more objectively reflect timbre discrimination thresholds in groups of CI and NH individuals. Note that, given its complexity, only a brief description of the protocol will be provided below (see Rahne et al., 2014 for the complete procedure). The task was an adaptive three-alternative forced-choice procedure in which just noticeable differences (JND) for temporal envelope modulation differences as well as spectral distribution differences were measured for each participant. Each participant's JND was then used to compute individual tone pairs, including (a) temporal envelope modulation/spectral distribution timbre discrimination and (b) above and below JND. Using these tone pairs, four oddball paradigms were created in order to elicit MMN. Specifically, Rahne et al. used the MMN amplitudes at the Fz electrode, representing the midline frontal area, which reflects one's ability to automatically detect acoustic change.

The article "Auditory Event-Related Potentials Associated With Music Perception in Cochlear Implant Users" was published in 2018. Journal: Front Neurosci.

First, the behavioral results showed that CI users' performance on spectral distribution and temporal envelope modulation were significantly lower than that of the NH controls. For CI users, a mean JND of 30.0 dB (TE tones in “good performers,” standard deviation [SD]: 8.6 dB) and 0.67 (S tones in all CI users, SD: 0.37) was found. For NH listeners, the mean JNDs were 7.2 dB (TE tone, SD: 4.7 dB) and 0.21 (S tones, SD: 0.28). Indeed, only four CI users out of fifteen were able to successfully complete the temporal envelope modulation condition. In terms of electrophysiological results, the authors report that both groups exhibited a significant MMN response in the above JND condition. However, no significant MMN response was found in the “below JND” condition—this for both groups. These results suggest electrophysiological measurements represent an effective way to evaluate timbre discrimination.

Overall, no difference was found between the CI and NH participants on the electrophysiological part of the study—which is coherent with the nature of the protocol, because the stimuli were adapted for each participant by being presented above or below their own just noticeable difference. In contrast, the CI users performed significantly worst than the NH controls on behavioral measures, which evaluated the discrimination of spectral distribution differences as well as temporal envelope modulation.

Indeed, the fact that the electrophysiological results can reveal the thresholds for both spectral distribution difference and temporal envelope modulation difference suggests that it might be an effective way to measure timbre discrimination in individuals whose understanding of the behavioral tasks, like prelingually deaf CI users, is more demanding. In sum, the study of Rahne et al. suggests that more complex protocols might be more effective to monitor timbre discrimination abilities than tasks that simply require participants to discriminate between musical instruments.

The article "Auditory Event-Related Potentials Associated With Music Perception in Cochlear Implant Users" was published in 2018. Journal: Front Neurosci.

It is important to emphasize here that studies do not consistently report altered timbre discrimination in CI users. For example, some studies have found no significant differences between CI users and NH controls on MMN amplitudes and/or latencies for saxophone timbre (standard stimulus: piano; deviant stimulus: saxophone), although significant differences were found for guitar timbre (standard stimulus: piano; deviant stimulus: guitar). These results suggest that, following implantation, some aspects of timbre discrimination might be preserved. Importantly, these studies have often used simple tasks in which timbre discrimination is easier or more obvious, thus allowing CI users to perform similarly to NH controls. However, when studies require participants to make more refined auditory analyses of the musical stimuli, the CI users usually experience more difficulties.

Overall, the present section seems to confirm that CI users experience difficulties with timbre perception, but also that the degree of their difficulties depends on the nature of the tasks that are used. More research needs to be done in order to better understand CI users' weaknesses and this has to be done with tasks that are demanding enough to better characterize CI users' difficulties with timbre perception.

### Perception of rhythm, tempo, meter, duration, and intensity

The behavioral studies that have investigated CI users' rhythm perception have shown that their perception of simple rhythm patterns is relatively good (Drennan and Rubinstein, 2008). Only one study has found that CI users perform significantly worse than controls on a rhythm task using a short inter-pulse interval in a six-pulse auditory pattern (Gfeller et al., 1997).

On the other hand, electrophysiological studies that have examined rhythm, tempo, meter, duration, and intensity of music in CI users have used multi-feature paradigms. For example, Sandmann et al. (2010) investigated musical sound perception in CI and NH individuals using an MMN paradigm. As mentioned earlier, the MMN component is elicited when an individual detects a different (or deviant) auditory stimulus among the “standard” stimuli that are presented. The MMN paradigm measured participants' ability to notice variations in music frequency, intensity, and duration. The task included different types of variations, namely, increments in frequency (493, 554, 622, and 698 Hz), decrements in intensity (61, 57, 53, 49 dB), and variations in stimuli duration (130, 110, 90, 70 ms). The results showed that, on deviations in duration, none of the groups showed a robust MMN response. However, the CI users exhibited MMN components of smaller amplitudes than the NH controls when exposed to variations in frequency and intensity. The CI users did not significantly differ from the NH controls when behavioral measures were used to examine variations in frequency, intensity, and duration of musical sounds [see Timm et al. (2014) for similar results].

The article "Auditory Event-Related Potentials Associated With Music Perception in Cochlear Implant Users" was published in 2018. Journal: Front Neurosci.

Thus, the above results suggest that CI users' ability to detect/notice variations in musical rhythm could be worse than that of NH individuals, which is consistent with the findings of behavioral studies showing that CI users experience difficulties with complex rhythm patterns.

### Musical meaning

It is interesting to reflect on the fact that songs often allow people to feel emotions, such as pleasantness. The cognitive ability that makes it possible to derive pleasantness from music has often been investigated in CI users. For example, Maglione et al., 2015) compared CI users and NH controls on the pleasantness that they felt while looking at a music video. The CI group was evaluated when they had only one implant and were evaluated again a few months later, after their second implantation. Perceived pleasure was assessed using an electroencephalogram measurement technique comparing the electrical activity in the different prefrontal areas (see Maglione et al., 2015 for the complete procedure). This technique made it possible to calculate an electrical imbalance index between left and right frontal regions while the participants were listening to the music video in three different conditions: (a) unmodified sound, (b) distorted sound, and (c) no sound. The results suggest that participants with bilateral implants experience a fluctuation in their perceived pleasures between the three different conditions similar to the variation found in the NH group (i.e., perceived pleasure: unmodified sound > distorted sound > no sound). Similar findings were found when the participants had only one implant.

A more recent procedure allows researchers to investigate relations between musical and lexical meaning. This procedure, which includes both behavioral and electrophysiological measures, consists in determining whether a musical stimulus is congruent or incongruent with a word (see Koelsch et al., 2004a for the detailed procedure). This word can be associated or not to the semantic sense of the musical piece an individual is listening to. For example, a fast musical except with a high pitch can easily be related to the word bird (i.e., related prime), but less to the word king (i.e., an unrelated prime). In terms of electrophysiological measurements, the procedure intends to elicit an N400 component. This component is an event-related brain potential that is related to meaning processing. Thus, it provides an objective evaluation of the congruence judgment of musical stimuli that the procedure entails (Koelsch et al., 2004a).

The article "Auditory Event-Related Potentials Associated With Music Perception in Cochlear Implant Users" was published in 2018. Journal: Front Neurosci.

A recent study has used this technique, including N400 measurements, in order to investigate CI users' comprehension/understanding of the meaning of music. Both pre-lingual CI users implanted before language acquisition (i.e., early childhood) and post-lingual CI users implanted after adolescence (i.e., long period of hearing deprivation before implantation) were included in this study. The results showed that the amplitude of the N400 component elicited by musical stimuli is positively and significantly correlated with the ability to make appropriate musical discriminations in NH individuals—but also in some CI users (Bruns et al., 2016). Indeed, an N400 was elicited in the post-lingual CI users, but not in the pre-lingual CI users. This is particularly relevant because it suggests that access to auditory input prior to deafness and, thus, to implantation is necessary to access the meaning of music.

## Discussion

The goal of the present short review was to identify the auditory event-related potential correlates underlying CI users' music perception. Reviewing the existing literature on CI users' music perception also highlighted the insufficient research on this topic and, accordingly, the scarcity of available evidence on the variables that might impact music perception in CI users. Moreover, the review shows that CI users' music perception can be measured objectively—with effective and demanding protocols. Indeed, the oddball paradigm was found to be an effective technique to measure CI users' perception of most fundamental musical features. Interestingly, the studies reviewed here clearly suggest that cochlear implantation alters most fundamental musical features, including pitch, timbre, melody perception, complex rhythm, and duration (e.g., Koelsch et al., 2004b; Timm et al., 2012, 2014; Zhang et al., 2013a,b; Limb and Roy, 2014). For a summary of how CI listeners fare on music perception tasks, see Table 1. In other words, the review confirms CI users' complaints about their reduced appreciation of music and, thus, stresses the importance of investigating the impact of deafness on music perception.

**Table 1:** Summary table of how CI listeners fare on music perception tasks.

**Study**	**Participants with CIs**	**Technique used**	**Musical traits examined**	**Results for CI users compared to the NH participants**	
Zhang et al., 2013b	*n* = 10 (3 F); Mean age = 53.6 years; Mean duration of profound deafness = 32.8 years	MMN	Pitch	One semitone	Rising:No MMN for CI only
					Falling:No MMN for CI only
				Five semitone	Rising:MMN elicited in 30% of CI users/ 80% for NH
					Falling:MMN elicited in 60% of CI users/ 80% for NH
Sandmann et al., 2009	*n* = 12 (10 F); Mean age = 44.3 years; Mean duration of profound deafness = 5.5 years	MMN	Pitch	N1 amplitude ↓	
				Altered hemispheric asymmetries	
Koelsch et al., 2004b	*n* = 12 (9 F); Mean age = 51.8 years; Mean duration of deafness = 11.8 years	ERAN	Timbre	3rd chord irregularity: No ERAN	
				5th chord irregularity: ERAN amplitude ↓	
		N5		3rd chord irregularity: No N5	
				5th chord irregularity: N5 amplitude ↓	
		MMN		MMN amplitude ↓	
Timm et al., 2012	*n* = 12 (8 F); Mean age = 45.3 years; Mean duration of deafness = 3.3 years	MMN	Timbre	Prolonged attack time: No MMN for CI users only	
				Shortened attack time: No MMN for CI users and NH	
				N1 amplitude ↓	
Zhang et al., 2013a	*n* = 12 (6 F); Mean age = 56.1 years; Mean duration of deafness = 35.5 years	MMN	Timbre	MMN peaks amplitudes ↓; latencies ↑	
Sandmann et al., 2010	*n* = 12 (6 F); Mean age = 55.3 years; Mean duration of deafness = 4.1 years	MMN	Frequency	MMN amplitude ↓	
			Intensity	MMN amplitude ↓	
			Duration	No MMN for CI and NH	
Maglione et al., 2015	*n* = 7	Imbalance index	Pleasantness	CI = NH	
Bruns et al., 2016	Pre-lingual: *n* = 15; mean age: 36 years; mean age at onset of profound hearing loss: 1.5 years	N400	Musical meaning	Pre-lingual CI users: No MMN	
	Post-lingual: *n* = 38 (21F); mean age = 65 years; mean age at onset of profound hearing loss: 56.6 years			Post-lingual CI users: MMN = NH	
Timm et al., 2014	*n* = 12 (7 F); Mean age = 43.6 years; Mean duration of profound deafness = 5.9 years	MMN	Pitch	Pitch violation:MMN amplitudes ↓; latencies ↑	
			Pitch	Pitch contour and violation:MMN amplitudes ↓; latencies ↑	
			Timbre	Guitar discrimination:MMN latencies ↑	
			Timbre	Saxophone discrimination:MMN elicited = NH	
			Intensity	MMN elicited = NH	
			Rhythm	No MMN for CI	

There are several limitations in the tasks that have been used and further studies should take them into consideration. A basic problem with interpreting the MMN studies is that there may be a perceptual contrast, but one does not necessarily know that the difference being perceived uses the same dimensions as the NH listener. For example, CI listeners could conceivably hear differences between musical instruments as changes in loudness, which will also produce an MMN. The studies need to probe not only the differences in performance, but also the perceptual dimensions that are involved. We know what those dimensions are for NH listeners, but they are ill-defined in the case of CI users. Also, further studies should probe MMN experiments with transposed melodies or chords. That would address issues related to pitch contours vs. musical intervals.

The article "Auditory Event-Related Potentials Associated With Music Perception in Cochlear Implant Users" was published in 2018. Journal: Front Neurosci.

Several other important points can be made from the above review. First, it is essential to properly investigate CI users' characteristics when evaluating their music perception. The quality of the acoustic signals provided by implants, the duration of deafness, and length of CI use are important variables that should be considered. Indeed, the studies reviewed differ greatly in terms of length of deafness. For example, the participants of Timm et al. (2014) and those of Zhang et al. (2013a,b) have a mean length of deafness of 5.93 and 35.5 years, respectively. It is, however, clear that length of deafness can greatly affect individuals' appreciation of music. Accordingly, Sandmann et al. (2010) found a significant negative correlation between duration of deafness and MMN responses for music frequency and intensity.

Although outside the scope of the present review, evidence shows that early cochlear implantation leads to better music perception than later cochlear implantation. Torppa et al. (2012) have investigated music perception in children with CIs. Interestingly, they found that the ERP activation patterns of children with CIs closely resembled that of normal hearing children—this on all musical dimensions, except intensity increment deviants. This further suggests that studies on CI users' musical perception abilities have to carefully control for the variables related to deafness and implantation.

Additional important variables to take into account include musical experience prior to implantation and number of implants. On the one hand, evidence shows that a background in musical perception prior implantation has a positive effect on music perception after implantation, making it possible to activate the concepts that are essential to access the meaning of music—as measured by the N400 protocol (Bruns et al., 2016). In terms of the number of implants, the few studies that have been done to date suggest that bilateral implantation has positive effects on music perception (Maglione et al., 2015). Studies must thus go further and contrast the music perception abilities of individuals with one implant to those of individuals with two implants (see Maglione et al., 2015 for an example). These studies would be helpful for clinicians who have to help patients decide whether or not they should get a second CI, by giving them arguments about the possible gains of bilateral implantation in terms of music perception. Further studies are, however, needed before any firm conclusion can be made on the positive impacts of bilateral implantation.

The article "Auditory Event-Related Potentials Associated With Music Perception in Cochlear Implant Users" was published in 2018. Journal: Front Neurosci.

The present review also highlights the importance of using complex electrophysiological protocols to examine CI users' complaints about music perception. Many of the studies reviewed above have used multi-feature paradigms that make it possible to investigate music perception rapidly and easily (e.g., Koelsch et al., 2004a,b; Sandmann et al., 2010; Timm et al., 2014). Adding this type of paradigm in routine evaluations of deaf individuals' music perception might eventually lead to a better understanding of the effectiveness of implants. Moreover, despite being rarely used, other electrophysiological protocols offer interesting knowledge on more complex musical features. For example, the imbalance index and the N400 are efficient electrophysiological techniques that make it possible to simultaneously evaluate several musical characteristics. The fact that they give information about several musical features at the same time make these measures particularly effective. Although more studies are needed before these techniques can be used in clinical contexts, they still make it possible to better understand musical perception in CI users.

## Conclusion

In summary, the presence of MMNs in CI users that are related to musical percepts indicates that they do possess some residual capacities for music perception after implantation. Although this gives hope for their future rehabilitation, there is still a substantial amount of work to do in order to improve CI users' music perception. As mentioned earlier, it is essential to determine which technique can be used to properly evaluate CI users' complaints about their music perception abilities. It is also important to better characterize the impact of their music perception complaints on their everyday life. To do so, paradigms measuring the pleasantness and/or the meaning of music appear to be particularly promising (see Bruns et al., 2016 and Maglione et al., 2015). As well, oddball and multi-feature paradigms were found to be particularly effective. It is, however, important to remember that multi-feature paradigms allow for more complete evaluations of musical perception abilities than oddball paradigms, which focus on more specific features.

Altogether, the present review suggests that cochlear implantation alters most fundamental musical features, including pitch, timbre, melody perception, complex rhythm, and duration (e.g., Koelsch et al., 2004b; Timm et al., 2012, 2014; Zhang et al., 2013a,b; Limb and Roy, 2014). Also, the results discussed here suggest that auditory event-related potentials are an effective technique to investigate CI users' music perception. Future studies using these techniques, however, need to take more variables into consideration, including prior musical training, duration of deafness, and number of implants.

The article "Auditory Event-Related Potentials Associated With Music Perception in Cochlear Implant Users" was published in 2018. Journal: Front Neurosci.

## Author contributions

AS wrote the first draft of the manuscript. AD and FC provided critical feedback to improve it.

### Conflict of interest statement

The authors declare that the research was conducted in the absence of any commercial or financial relationships that could be construed as a potential conflict of interest.
